# The Clinical Effects of the Phlegm-Resolving Method in the Treatment of Obstructive Sleep Apnea-Hypopnea Syndrome: A Meta-Analysis of Randomized Controlled Trials

**DOI:** 10.1155/2022/7426552

**Published:** 2022-07-31

**Authors:** Sifeng Zhou, Haishu Xu, Juan Liu, Xinsheng Fan

**Affiliations:** ^1^School of Traditional Chinese Medicine·Integrated Chinese and Western Medicine, Nanjing University of Chinese Medicine, Nanjing, Jiangsu 210023, China; ^2^Department of Endocrinology, Rudong Hospital of Traditional Chinese Medicine, Nantong, Jiangsu 226400, China; ^3^Department of Pharmacy, Rudong Hospital of Traditional Chinese Medicine, Nantong, Jiangsu 226400, China

## Abstract

**Objective:**

This study evaluated the clinical efficacy and safety of the phlegm-resolving method in traditional Chinese medicine (TCM) for the treatment of obstructive sleep apnea-hypopnea syndrome (OSAHS).

**Methods:**

We searched the PubMed, Embase, Cochrane Library, Wanfang, CNKI, and VIP databases according to specific search strategies. The data were analyzed using RevMan 5.3 software.

**Results:**

Thirteen randomized controlled trials (RCTs) comprising 882 patients with OSAHS were selected. Compared to continuous positive airway pressure (CPAP), the phlegm-resolving method of TCM combined with CPAP significantly more effectively improved the apnea/hypopnea index (AHI), Epworth Sleepiness Scale (ESS), and lowest oxygen saturation (LSaO_2_). While the treatment effect was better for a treatment duration of >6 weeks compared to that at ≤6 weeks, the difference was not statistically significant. Compared to health guidance alone, the combination of the phlegm-resolving method in TCM with health guidance showed significantly better efficacy in improving AHI, ESS, and LSaO_2_. In terms of reducing ESS and increasing LSaO_2_, the effect was better for treatment courses >6 weeks. When the AHI was reduced, a duration of ≤6 weeks showed more advantages; however, the difference was not significant. Only one study reported mild nausea in one participant in the treatment group at the initial stage of treatment; the remaining studies did not mention any side effects.

**Conclusion:**

Both the resolving phlegm method of TCM combined with CPAP and the resolving phlegm method of TCM combined with health guidance were more effective in improving AHI, LSaO_2_, and ESS compared to the control group.

## 1. Introduction

Obstructive sleep apnea-hypopnea syndrome (OSAHS) is a disorder caused by upper respiratory tract stenosis that is characterized by sleep apnea, hypopnea, microarousal, and sleep fragmentation [1]. Chronic intermittent hypoxia (CIH) is the main pathophysiological manifestation of OSAHS, leading to repeated hypoxia and reoxygenation of organs, which further causes inflammation and oxidative stress [2]. It is currently considered to be related to various diseases, such as hypertension, diabetes, stroke, cardiovascular disease (CVD), and cancer [3–8]. The prevalence of OSAHS in men is higher than that in women. The common risk factors include hypothyroidism, tonsil hypertrophy, obesity, alcohol consumption, and nasal obstruction [9]. With improvements in living standards, the global incidence of OSAHS is also increasing annually, with approximately 25% of men and 13% of women experiencing OSAHS worldwide [10]. Owing to excessive drowsiness, irascibility, reduced concentration and memory, lack of vigor, and erectile dysfunction, many patients have varying degrees of depressive symptoms, which seriously affect their physical and mental health [11, 12].

At present, overnight polysomnography (PSG) is considered the gold standard for the diagnosis of OSAHS. Considering the series of complications of OSAHS, diagnosed patients should be treated effectively and immediately. Given the high incidence of OSAHS, many treatments have been proposed to improve the disease. In recent decades, nasal continuous positive airway pressure (nCPAP) therapy has resulted in significantly reduced OSAHS complications and mortality [13]. nCPAP is the preferred treatment for patients with symptomatic OSAHS because of its significant effects in managing apnea, eliminating hypoxia, improving sleep quality, and reducing the incidence of cardiovascular diseases [14]. Recent data confirm that nCPAP not only reduces blood pressure [15], but also improves blood glucose and lipid metabolism [16, 17]. Oral appliances may be an alternative for patients unwilling to receive CPAP treatment or who have failed to adhere to CPAP treatment. Surgery may also be recommended for patients with large palatine or tonsillar hypertrophy [18].

Although evidence has demonstrated the significant effect of CPAP on OSAHS, due to its discomfort and limitations, many patients have difficulty continuing CPAP or seek complementary and alternative therapies [19]. Surgery and oral appliances cannot be used on a large scale because of their obvious side effects. Therefore, finding safe and effective alternative treatments is of great significance. traditional Chinese medicine (TCM) is a medical system with a history spanning thousands of years. The many methods of curing diseases in TCM include herbal medicine, acupuncture, and massage. OSAHS is called “snoring disease” in Chinese medicine. Its pathogenesis includes disturbance of zang-fu organs, disordered qi movement, phlegm accumulation, and blood stasis, which lead to airway obstruction. Oral herbal medicines, acupuncture, and auricular point pressure therapies are often used to treat OSAHS. Acupuncture is also effective in treating patients with OSAHS [20]. Some articles have also confirmed the effectiveness of Chinese herbal medicines in the treatment of OSAHS [21]. However, no meta-analysis has been reported on the treatment of OSAHS using the phlegm-resolving method in TCM. Owing to the lack of high-quality evidence-based medicine, the mainstream medical community has not yet recognized the efficacy of Chinese herbal medicine in OSAHS. Therefore, the present study evaluated the therapeutic effect of resolving phlegm in OSAHS, which may be a simple and inexpensive treatment for OSAHS.

## 2. Materials and Methods

### 2.1. Literature Search

This meta-analysis conformed to the preferred reporting items for systematic reviews and meta-analyses (PRISMA) guidelines [22]. We systematically searched the PubMed, EMBASE, Cochrane Library, Wanfang, CNKI, and VIP electronic databases from the establishment of the databases to February 2021. All relevant bibliographies were manually searched, regardless of the language. We adopted a search strategy of combining medical subject headings (MeSH) with free terms, and searched for as many qualified studies as possible.

The search terms were: (“Sleep Apnea, Obstructive” or OSAHS or obstructive sleep apnea or sleep apnea or sleep hypopnea or obstructive sleep apnea-hypopnea syndrome) and (“resolving phlegm method” or “dissipating phlegm method” or “reduce phlegm” or “huatanfa”).

### 2.2. Inclusion and Exclusion Criteria

We applied the PICOS (participants, interventions, comparisons, outcomes, and study design) principle for our inclusion and exclusion criteria. All enrolled patients were diagnosed with OSAHS by PSG. There were no restrictions on sex and race, and all participants were adults. All subjects in the treatment groups primarily received Chinese medicine, mainly Chinese herbal medicine for resolving phlegm. The subjects allocated to the control groups received health guidance or CPAP treatment. The chief outcome in this study was AHI, while LSaO_2_ and ESS were the secondary outcomes. We included only randomized controlled trials (RCTs). Animal experiments, acupuncture or other external treatments, reviews, case reports, and duplicate studies were excluded.

### 2.3. Data Extraction

Two reviewers (Sifeng Zhou and Juan Liu) independently reviewed all the included papers, with each unaware of the other's findings. Two reviewers extracted and collected the original data independently, which including basic information on the included research, study methodological content, interventions, and outcome indicators. Any uncertainties or disagreements were resolved through discussion within the group or with a third researcher (Xinsheng Fan) until consensus was reached.

### 2.4. Risk of Bias Assessment

We evaluated the quality of the included articles using the Cochrane Evaluation Manual Handbook, which considers seven items: random sequence generation, allocation concealment, blinding of participants and personnel, blinding of outcome assessment, incomplete outcome data, selective reporting, and other sources of bias. Two researchers independently assessed each study according to the criteria for risk of bias as low, high, and unclear.

### 2.5. Data Statistics and Analysis

We used RevMan 5.3 software to conduct this meta-analysis. As all outcome indicators included in this study were continuous variables, the mean differences (MDs) and related 95% confidence intervals (CIs) for AHI, LSaO_2_, and ESS were calculated. The Higgins *I*^2^ test was used to calculate the heterogeneity of all enrolled studies (*I*^2^ < 50% suggested satisfactory heterogeneity). When the heterogeneity among studies was obvious, a random-effects model was used to analyze the data; otherwise, a fixed-effects model was used. A funnel plot was constructed to detect potential publication bias when the number of included studies was >10.

## 3. Results

### 3.1. Literature Search

The flow of the literature selection is summarized in Figure 1. In total, 592 articles were retrieved, including 269 from CNKI, 232 from Wanfang, and 91 from VIP. A total of 336 duplicate papers were excluded. A further 297 RCTs were excluded after browsing the titles and abstracts. After screening the full texts of the remaining 39 studies, seven articles were excluded due to duplication, three papers were excluded for lack of detail on the composition of the prescription, another three articles were excluded because they did not provide complete basic information on the included population, and 13 reports were excluded because they did not provide primary and secondary outcomes. Finally, 13 articles [23–35] met the inclusion criteria for this meta-analysis.

### 3.2. Features of Selected Studies

This study analyzed 13 RCTs with 882 patients with OSAHS, including 441 patients each in the treatment and control groups, respectively. These RCTs were published between 2012 and 2019, and all were conducted in China, with a minimum sample of 39 cases and a maximum sample of 100 cases. The treatment duration ranged from 20 days to 3 months. One study [33] included only patients with mild to moderate disease, and one study [35] included only patients with moderate-to-severe disease. Hu et al. [23]separately reported mild and moderate-to-severe patients. In addition, no studies observed any distinct differences in indices between the two groups before treatment. The baseline information of all enrolled studies is presented in Table 1. The treatment methods used in the trials are listed in Table 2.

### 3.3. Risk of Bias Assessment

The Cochrane Evaluation Manual Handbook was used to evaluate the risk of bias in the selected papers. All selected trials reported randomization. However, only nine trials [23, 25–29, 31, 34, 35] performed random sequence generation, eight of which [23, 25–29, 31, 35] used random number tables and one of which [34] used computer-generated random codes for random allocation. Only one study described allocation concealment [26], and no studies were blinded. All anticipated indices were described in the included articles and none were terminated early. The methodological quality assessments are listed in Table 3. The risk of bias assessment for each study is summarized in Figure 2.

### 3.4. Meta-Analysis Results

As the medication course may affect the treatment effect, subgroup analyses were performed accordingly.

#### 3.4.1. Phlegm-Resolving Method in TCM Combined with CPAP versus CPAP

*AHI*. Eight studies [23, 27–30, 32, 34, 35] reported AHI as the outcome. Among them, six studies [23, 27–29, 34, 35] achieved a remedy duration of ≤6 weeks, while two studies [30, 32] had a treatment course of >6 weeks. Because obvious heterogeneity was observed among these studies, we adopted a random-effects model to analyze the data. Compared to the control group, ≤6 weeks (−8.29 (−12.09, −4.49)) and >6 weeks (−8.36 (−18.79, 2.06)) significantly improved AHI. The curative effect on AHI of the treatment group with a remedy duration of >6 weeks was better than that of ≤6 weeks, but the difference was not statistically significant (*P*=0.99), suggesting that the effect of different treatment courses on AHI was not obvious (Figure 3).

LSaO_2._ Five studies [23, 27, 29, 34, 35] measured LSaO_2_ as an outcome. None of the patients had a treatment course >6 weeks. Because we found obvious heterogeneity among the studies, a random-effects model was adopted. The results explained that compared to the control group, although the treatment course was ≤6 weeks (10.42(1.62, 19.22)), the phlegm-resolving method in TCM combined with CPAP significantly increased LSaO_2_ (Figure 4).

ESS. Five studies [23, 29, 30, 34, 35] measured ESS as an outcome. Only one study [30] carried out a treatment course >6 weeks. Due to the significant heterogeneity, we applied the random-effects model. The results demonstrated that compared to the control group, although the treatment course was ≤6 weeks (−2.30 (−3.72, −0.88)), the phlegm-resolving method in TCM combined with CPAP further improved the ESS (Figure 5).

#### 3.4.2. Phlegm-Resolving Method in TCM Combined with Health Guidance versus Health Guidance

*AHI.* Six studies [23–26, 31, 33] measured AHI as an outcome. Two studies [23, 33] carried out a treatment duration of ≤6 weeks; the other studies had courses >6 weeks. As no heterogeneity was observed among the included trials (*I*^2^ = 0), the fixed-effects model was adopted. Compared to the control group, the treatment group showed further improvement in AHI regardless of whether the course of treatment was ≤6 weeks (−5.23(−7.35, −3.11)) or > 6 weeks (−5.70(−10.15, −1.25)). The treatment effect on AHI for a duration of >6 weeks was better than that of ≤6 weeks; however, the difference was not statistically significant (*P*=0.85) (Figure 6).

LSaO_2._ Five studies [23–25, 31, 33] measured the LSaO_2_ as an outcome assessment. Two of these studies [23, 33] had a treatment course ≤6 weeks, while the other three [24, 25, 31] had a course of >6 weeks. Owing to obvious heterogeneity, we employed a random-effect model. Compared to the control group, the phlegm-resolving method in TCM combined with health guidance more effectively improved LSaO_2_. Compared to the course of treatment ≤6 weeks (5.06(0.40, 9.71)), the effect was better when the course of treatment was >6 weeks (7.04(4.87, 9.21)); however, the difference was not statistically significant (*P*=0.45) (Figure 7).

Five studies [23–26, 33] recorded ESS in the trials, two of which [23, 33] conducted treatment courses ≤6 weeks; the remaining three [24–26] were >6 weeks. Since the calculation results showed that *I*^2^ < 50%, we applied a fixed-effects model for the meta-analysis. The results showed that compared to health guidance alone, health guidance combined with the phlegm-resolving method in TCM significantly improved ESS regardless of the treatment course. When the treatment course was >6 weeks (−1.45(−2.22, −0.68)), the curative effect was better than that of ≤6 weeks(−1.15(−1.96, −0.35)), but the result was not statistically significant (*P*=0.61) (Figure 8).

### 3.5. Adverse Events

Six studies [24–26, 32–34] reported safety evaluations, among which only one study [25] reported mild nausea in one participant in the treatment group during the initial stage of treatment. The remaining studies did not mention any side effects, indicating that the phlegm-resolving method in TCM is safe for the treatment of OSAHS.

### 3.6. Publication Bias

Due to the insufficient number of covered studies, publication bias was not evaluated. However, a potential publication bias cannot be ruled out.

## 4. Discussion

At present, PSG remains the gold standard for the diagnosis of OSAHS. The severity of this condition is classified according to AHI and LSaO_2_. The ESS is a simple, self-administered questionnaire used to assess patients' daytime sleepiness. The outcome indices in our study were AHI, LSaO_2_, and ESS. Both AHI and LSaO_2_ can be measured directly by PSG, while the ESS was scored by the participants themselves. The therapeutic effect was presented intuitively using these three indicators. Given that treatment duration may affect outcomes, a subgroup analysis was performed.

This study systematically and objectively evaluated the efficacy and advantages of the phlegm-resolving method in TCM for the treatment of OSAHS, providing a strong theoretical basis for the use of TCM in OSAHS prevention and treatment. The results of our meta-analysis showed that both CPAP and health guidance can improve AHI, LSaO_2_, and ESS; however, they can achieve better results when combined with the phlegm-resolving method in TCM. Moreover, compared to CPAP, the phlegm-resolving method of TCM combined with CPAP significantly more effectively reduced AHI and ESS and increased LSaO_2_. While the treatment effect was better for treatment durations >6 weeks, the difference was not statistically significant. Compared to health guidance alone, the phlegm-resolving method in TCM combined with health guidance showed significantly better efficacy in diminishing AHI and ESS and enhancing LSaO_2_. The effect of reducing AHI and ESS and increasing LSaO_2_ was better when the treatment course was >6 weeks, but the difference was not statistically significant. A longer treatment duration may be required to obtain more significant differences. Our meta-analysis included 13 RCTs with 882 patients, none of whom experienced serious adverse events associated with the phlegm-resolving method of TCM. These findings indicate that the phlegm-resolving method in TCM is effective and safe for the treatment of OSAHS and can be used as a potential alternative therapy for OSAHS.

The therapeutic purpose of OSAHS is to reduce AHI, increase LSaO_2_, improve sleep disorders, and improve patient quality of life. The treatment methods for OSAHS mainly include CPAP, oral appliances, and surgical treatment [36], and there are currently no effective drugs for treatment [37]. Many patients have difficulty adhering to CPAP treatment due to its inconvenience and discomfort. Oral appliances and surgical treatment are difficult to widely promote due to the high economic burden and pain. Therefore, new treatments are urgently required for OSAHS. TCM is a complementary and alternative therapy with remarkable curative effects, high safety, and fewer adverse reactions. While there is no record of the name OSAHS in Chinese medicine, according to its symptoms, OSAHS can be classified as sleepiness, snoring, and other related diseases. According to TCM theory, the main pathogenic factors of OSAHS are phlegm and dampness [38]. Therefore, the phlegm-resolving method in TCM was mainly used in the treatment groups included in this meta-analysis. This method aims to gradually resolve and eliminate phlegm by targeting the etiology and pathogenesis of all phlegm syndromes. The resolving phlegm method is used in combination with related treatment methods, including methods of exterior-relieving, warming yang, dispelling stasis, tonifying the kidney, nourishing yin, and regulating Qi. Our meta-analysis is the first to assess the efficacy of the phlegm-resolving method in TCM in OSAHS based on 13 studies comprising 882 subjects. Our results confirmed that the resolving phlegm method in TCM had satisfactory effectiveness and safety in OSAHS. Moreover, subgroup analysis showed a positive correlation between efficacy and the duration of treatment, although more studies are needed to confirm the significance of this relationship. However, when the treatment course is too long, the treatment effect may be affected by factors such as compliance.

However, this study has some limitations. First, the sample size of most enrolled trials was small and the quality was unsatisfactory. Second, all the selected trials were conducted in China, which may have been subject to publication bias. Third, most studies failed to address blinding, which may have affected the objectivity of the results. Fourth, due to uncertainty in the composition of TCM prescriptions, although the studies we included were mainly based on the treatment of phlegm-resolving methods, the Chinese herbal medicines differed among studies, which led to some potential bias in our research. Fifth, different types of Chinese medicines, different decoction methods, and even different times of taking the medicine, which can affect their efficacy, might be another source of bias. Finally, because the resolving phlegm method includes a variety of treatment methods, the intervention methods are correspondingly broad, which leads to high inter-study heterogeneity. Therefore, more strictly designed, multicenter, large-sample RCTs are needed to provide higher-quality evidence.

## 5. Conclusion

In summary, the results of our meta-analysis indicated that both phlegm-resolving TCM combined with CPAP and phlegm-resolving TCM combined with health guidance significantly improved AHI, LSaO_2_, and ESS. The subgroup analysis also suggested that the therapeutic effect of the phlegm-resolving method of TCM on OSAHS was related to the course of treatment but may also be affected by compliance, the environment, and other factors. In consideration of the treatment courses for comparison, it might be impossible to draw accurate conclusions due to sample size, compliance, and other reasons. More rigorously designed RCTs with larger sample sizes are required.

## Figures and Tables

**Figure 1:** Flowchart of the literature search.

**Figure 2:** Risk of bias diagram.

**Figure 3:** Forest plot of the phlegm-resolving method in traditional Chinese medicine (TCM) combined with continuous positive airway pressure (CPAP) versus CPAP: apnea/hypopnea index (AHI).

**Figure 4:** Forest plot of the phlegm-resolving method in traditional Chinese medicine (TCM) combined with continuous positive airway pressure (CPAP) versus CPAP: lowest oxygen saturation (LSaO_2_).

**Figure 5:** Forest plot of the phlegm-resolving method in traditional Chinese medicine (TCM) combined with continuous positive airway pressure (CPAP) versus CPAP: Epworth sleepiness scale (ESS).

**Figure 6:** Forest plot of the phlegm-resolving method in traditional Chinese medicine (TCM) combined with health guidance versus health guidance: apnea/hypopnea index (AHI).

**Figure 7:** Forest plot of the phlegm-resolving method in traditional Chinese medicine (TCM) combined with health guidance versus health guidance: lowest oxygen saturation (LSaO_2_).

**Figure 8:** Forest plot of the phlegm-resolving method in traditional Chinese medicine (TCM) combined with health guidance versus health guidance: epworth sleepiness scale (ESS).

**Table 1:** Baseline information of the enrolled studies.

Study	Sex (M/F)		Population		Age(mean or range)		Duration oftreatment	Mainoutcome
	*T*	*C*	*T*	*C*	*T*	*C*		
Hu et al., 2012 [23]	17/2	18/2	19	20	50.4 ± 12.8	51.4 ± 14.1	30 days	AHI, LSaO_2_, ESS
Wang et al., 2013 [24]	32/8	36/4	40	40	47.02 ± 14.24	43.63 ± 12.16	3 months	AHI, LSaO_2_, ESS
Chen et al., 2015 [25]	20/10	21/9	30	30	68.2 ± 5.9	65.0 ± 6.3	12 weeks	AHI、LSaO_2_、ESS
Feng et al., 2015 [26]	26/4	27/3	30	30	43.34 ± 6.42	42.19 ± 7.49	12 weeks	AHI, ESS
Lv et al., 2017 [27]	19/6	20/5	25	25	52.5 ± 5.4	51.2 ± 5.1	20 days	AHI, LSaO_2_
Liu et al., 2017 [28]	26/6	23/9	32	32	46.3 ± 2.2	47.5 ± 3.6	1 months	AHI
Gui et al., 2017 [29]	21/29	20/30	50	50	54.19 ± 4.26	54.26 ± 3.19	4 weeks	AHI, LSaO_2_, ESS
Yin et al., 2017 [30]	34/11	33/12	45	45	52.49 ± 3.27	52.68 ± 3.59	3 months	AHI, ESS
Xu et al., 2018 [31]	22/6	23/4	28	27	42.80 ± 11.94	43.72 ± 13.96	12 weeks	AHI, LSaO_2_
Lu, 2018 [32]	38/2	39/1	40	40	43.19 (35–58)	42.86 (32–55)	8 weeks	AHI
Jin et al., 2019 [33]	20/8	21/7	28	28	42.25 ± 13.60	43.11 ± 12.09	1 months	AHI, LSaO_2_, ESS
Yang et al., 2019 [34]	32/8	34/6	40	40	40.2 ± 10.1	41.3 ± 11.4	30 days	AHI, LSaO_2_, ESS
Liu et al., 2019 [35]	20/12	22/10	32	32	58.1 ± 5.0	59.0 ± 5.0	4 weeks	AHI, LSaO_2_, ESS

Note. *M*, male; *F*, female; *T*, treatment group; *C*, control group; N.R, not reported.

**Table 2:** Treatment methods used.

Study	Dosage form	Intervention	
		*T*	*C*
Hu et al., 2012 [23]	Decoction	Mild: phlegm-eliminating and snore-stoppingdecoction + health guidance Moderate and Severe: phlegm-eliminatingand snore-stopping Decoction + CPAP + healthguidance	Mild: Health guidance Moderate and severe:CPAP + health guidance
Wang et al., 2013 [24]	Granule	Erchen snoring Granule + health guidance	Health guidance
Chen et al., 2015 [25]	Granule	Jiawei ditan decoction + health guidance	Health guidance
Feng et al., 2015 [26]	Decoction	Jianpi huatan formula + health guidance	Health guidance
Lv et al., 2017 [27]	Decoction	Huatan Zhihan decoction + CPAP + health guidance	CPAP + Health guidance
Liu et al., 2017 [28]	Decoction	Snoring I + CPAP	CPAP
Gui et al., 2017 [29]	Decoction	Modified huatan quyu kaiqiaodecoction + CPAP + health guidance	CPAP + Health guidance
Yin et al., 2017 [30]	Decoction	Jianpi Huatan decoction + CPAP + health guidance	CPAP + Health guidance
Xu et al., 2018 [31]	Granule	Erchen snoring granule + health guidance	Health guidance
Lu, 2018 [32]	Decoction	Modified erchen decoction + CPAP	CPAP
Jin et al., 2019 [33]	Granule	Xiaohan Liqi granules + health guidance	Health guidance
Yang et al., 2019 [34]	Decoction	Modified erchen decoction and taohong siwudecoction + CPAP + health guidance	CPAP + Health guidance
Liu et al., 2019 [35]	Decoction	Quyu Huatan decoction + CPAP + health guidance	CPAP + Health guidance

Note. *T*, treatment group; *C*, control group; N.R, not reported; CPAP, continuous positive airway pressure.

**Table 3:** Assessment of methodological quality.

Study	Random method	Allocation concealment	Blinding	Drop out/Withdrawal	Selective reporting	Other biases
Hu et al., 2012 [23]	R.N.T	N.R	N.R	None	Yes	Unclear
Wang et al., 2013 [24]	N.R	N.R	N.R	None	Yes	Unclear
Chen et al., 2015 [25]	R.N.T	N.R	N.R	None	Yes	Unclear
Feng et al., 2015 [26]	R.N.T	Yes	N.R	None	Yes	Unclear
Lv et al., 2017 [27]	R.N.T	N.R	N.R	None	Yes	Unclear
Liu et al., 2017 [28]	R.N.T	N.R	N.R	None	Yes	Unclear
Gui et al., 2017 [29]	R.N.T	N.R	N.R	None	Yes	Unclear
Yin et al., 2017 [30]	N.R	N.R	N.R	None	Yes	Unclear
Xu et al., 2018 [31]	R.N.T	N.R	N.R	Drop out: 5	Yes	Unclear
Lu, 2018 [32]	N.R	N.R	N.R	None	Yes	Unclear
Jin et al., 2019 [33]	N.R	N.R	N.R	Drop out: 4	Yes	Unclear
Yang et al., 2019 [34]	Java random number	N.R	N.R	None	Yes	Unclear
Liu et al., 2019 [35]	R.N.T	N.R	N.R	None	Yes	Unclear

Note. N.R, not reported; R.N.T, random number table.

## Data Availability

All data are available in this study.
